# Construction of Enterprise Financial Early Warning Model Based on Logistic Regression and BP Neural Network

**DOI:** 10.1155/2022/2614226

**Published:** 2022-05-24

**Authors:** Jincheng Lyu

**Affiliations:** Tianjin Xiqing Economic Development Co., Ltd., Tianjin 300380, China

## Abstract

At present, the number of enterprises in financial crisis in China is rising sharply, and the ability of enterprises to resist risks is generally weak. Therefore, it is necessary to establish a corporate financial crisis early warning system, to detect the signs of corporate financial crisis before it arrives and to inform managers in advance, so that effective measures can be taken as soon as possible to eliminate hidden dangers. This paper selects the two-year data of 40 companies from 2017 to 2019 as training samples and the data of 20 companies as prediction samples. After testing, 12 index variables that can reflect the financial problems of energy companies are finally selected as the basis for modeling. Then, we use Logistic and BP neural network modeling, respectively, to study and compare the data from 2017 to 2019 to predict the financial risk in the following year. The results show that the BP neural network model in the two models is better than the Logistic model in terms of fitting degree or prediction accuracy for enterprise financial early warning. Therefore, the BP neural network model has a better effect and is more suitable for the practical application of enterprises in China.

## 1. Introduction

With the rapid development of the economy in China, small- and medium-sized enterprises, as the most vital group in China, have grown into an important part of the economy, whether in foreign export trade or in increasing employment opportunities and increasing GDP. At present, China has 10 million industrial and commercial registered enterprises, of which 99% are small- and medium-sized enterprises. Small- and medium-sized enterprises provide 80% of the urban population's employment, and 70% of innovation comes from small- and medium-sized enterprises. In the competitive environment dominated by the buyer's market, the market competition continues to intensify [1–3]. In order to consolidate or expand their competitive advantages, small- and medium-sized enterprises in the industry must provide customers with competitive products and services, including preferential credit settlement methods, mainly in the form of credit sales. However, this method will make the enterprise itself bear the risk of the other party's use, which often causes the accounts receivable to be unable to be recovered in full and on schedule, and many enterprises fall into the dilemma of “not selling on credit and waiting to die and selling on credit to court death.” This requires enterprises to fully understand their customers, develop a reasonable financial system, and lock down the financial risks of the enterprise by conducting financial early warning assessments of their finances before cooperating [4–7].

Although small- and medium-sized enterprises have made significant contributions to the economic growth in China, due to their lack of strict accounting systems, lack of professional financial personnel, and relatively small scale, it is currently difficult for small- and medium-sized enterprises to obtain financing with high financing costs to obtain financing from financial institutions. At this stage, banks, other enterprises, and financial institutions do not have a reasonable financial early warning system to assess the financial risks and experience of SMEs, and they will not easily lend to SMEs. The problem of shortage of funds has limited the development of enterprises to a certain extent [8–10].

Since the 1930s, many scholars have devoted a lot of time and energy to the study of financial crisis early warning and have also developed some more objective, rigorous, and at the same time simple and feasible assessment methods. Fitzpatrick (1932) studied a sample of 19 firms and used a single financial ratio to divide the sample into bankrupt and nonbankrupt groups. It is found that net profit/shareholders' equity and shareholders' equity/liabilities have a good ability to discriminate financial crisis, and these two ratios show significant differences in the first three years of operating failure. Secrist (1938) used the ratio of assets/liabilities to compare the difference between failed banks and normal banks [11–13]. The research of Fitz et al. is still in the stage of descriptive analysis, and in the following 20 years, there has been no significant progress in the study of financial crisis prediction. After 1990, related research began to change from simply studying corporate financial variables to predict corporate financial risks, to adding variables such as macroeconomic environment to the study for further research. In the subsequent series of studies, some scholars such as Odom and Coats tried to use the artificial neural network (ANN) to conduct research. From the obtained results, the success rate is relatively low. Only Coats (1993) used Altman to discriminate on the basis of the five judgment variables proposed by the *Z*-Score model and obtained relatively good judgment results in the prediction of crisis enterprises. The accuracy rate is 91%, and the accuracy rate for normal enterprise prediction is 96%, which is slightly better than the discriminant analysis model. So far, the research on financial early warning in China is not very sufficient, and it is basically in its infancy [14–17]. Among the scholars who studied, most of them introduced foreign theories in terms of research in their own countries. Some of them discussed theories and feasibility and put forward suggestions and measures in system construction and legislation, and very few conducted in-depth research on issues such as models.

This paper selects the financial indicator data of 60 companies from 2017 to 2019 and divides it into training samples and prediction samples for empirical research. We use the SPSS20.0 software to screen out model indicators for the next step of model building, optimize variables by factor analysis, preprocess the data, and establish and compare Logistic models using financial indicators and adding nonfinancial indicators. Matlab software is used to train the training samples to establish a BP neural network early warning model, and the prediction samples are used to test the accuracy of the model prediction [18–20].

## 2. Methods and Theory

### 2.1. Design Steps

The structure of the financial early warning model can be divided into five steps as shown in Figure 1. First, we determine the research sample type. The financial early warning has certain limitations. Different periods and different industries will correspond to different financial characteristics. Determining the sample type and enterprise characteristics is research. The second step is to select index variables according to the characteristics of different industries and adjust them appropriately. Third, we need to screen the financial indicators and select the indicators required to build the model. The screening methods in existing research generally include factor analysis and principal component analysis method. Fourth, we establish the model. This paper uses Logistic regression and BP neural network model to establish financial early warning models, respectively, to evaluate the warning level.

### 2.2. Logistic Early Warning Model Design

#### 2.2.1. Research Sample

In this paper, 60 companies from 2017 to 2019 are selected first, and the sample companies are screened and classified according to the classification standard of early warning degree. When classifying the sample data, we try to maintain the balance between the samples. The specific classification is shown in Table 1.

#### 2.2.2. Early Warning Indicator Variables

Preliminary selection is made from two aspects: financial indicators and nonfinancial indicators. Financial indicators are selected from five aspects: profitability and income quality, solvency and capital structure, operating capacity and cash flow, development capacity, and risk level. Nonfinancial indicators include related party transactions, violations, audit reports, litigation, and arbitration. We select indicators that can truly reflect the financial risks of the industry and then conduct further screening. Through the normality test of the indicators and the significance test, the indicators selected in this paper are shown in Table 2.

Factor analysis requires a high degree of correlation between variables, and a correlation test needs to be carried out before factor analysis. Financial indicators are calculated through financial data, and there is a high degree of correlation between variables. Nonfinancial indicators do not need factor analysis, so we incorporate it directly into the variables of the final model building.

Through the factor analysis method of the KMO and Bartlett sphere test, 11 financial indicators are preliminarily screened to ensure that the screened financial variables are suitable for the empirical requirements of companies. The data are obtained through SPSS analysis software to obtain the 11 indicators for factor analysis. Through factor analysis, it is concluded that the eigenvalues of the first four common factors exceed 1, so the first four common factors can be used as surrogate variables for 11 financial indicators. The public factor Fl can be explained by variables 3, 4, 5, and 6, reflecting the solvency and capital structure. The public factor F2 can be explained by 1, 2, 9, and 10, reflecting the profitability and growth ability. The public factor F3 can be explained by variables 7 and 8, reflecting the level of operating capacity and cash flow. The public factor F4 can be explained by variable 11, reflecting the risk level of the enterprise.

#### 2.2.3. BP Neural Network Early Warning Model Design

The realization of the BP neural network financial crisis early warning model is divided into input and output layer variable design, hidden layer node design, error and learning rate selection, etc. The realization process is as follows:

(1) *Select Training and Prediction Samples*. According to the research direction, the financial samples of enterprises are selected, the two-year financial data of 40 companies are used as training samples for training, the data of 20 companies are used for prediction, and the predicted value of the model is compared with the expected output value.
(2) *Determine the Input and Output Layer Changes*. In general, the number of input nodes is positively correlated with the approximation result of the neural network. The more input neuron nodes, the better the approximation effect. However, when irrelevant indicators are incorporated into the neural network training, the fitting will occur due to the increase in the number of indicators. Too many nodes will increase the calculation amount of the BP neural network, which will lead to longer model training time, affecting the output results.
  According to the indicator variables selected by the Logistic early warning model, 11 financial indicators and 1 nonfinancial indicator are used as the input vectors of the model and the number of input variables is confirmed; that is, the input layer of the model is positioned as 12 in this paper.
  The output layer uses the expected output value after training and the classification result of the financial warning degree of energy enterprises as the output vector for training. Some studies have concluded that the number of nodes in the prediction output layer of the financial crisis is set to 1.
(3) *Determine the Number of Hidden Layer Nodes*. The model is more complicated to determine the number of nodes in the hidden layer, which is generally set by empirical values. According to the comprehensive consideration of the sample size and the number of variables, setting the appropriate number of nodes is directly related to the results of the model. Too many hidden layer nodes will increase the learning practice, and too few will reduce the collection ability, and it is impossible to find the inherent laws of the data through self-learning.

The number of hidden layer nodes is different for different models, and the following are selected from common empirical formulas, where *n* is the number of input nodes and *m* is the number of output nodes:

(1) $$\begin{array}{c} L={\text{log}}_{2}n, \end{array}$$

(2) $$\begin{array}{c} L=\sqrt{m+n}+a, \end{array}$$

(3) $$\begin{array}{c} L=n+0.618\left(n-m\right). \end{array}$$

In this paper, a is a constant between 1 and 10. Empirical formula (2) is selected. First, the input node *n* = 12 is brought into the model, and a tentative test is carried out, and it is continuously adjusted according to the results. The final number of nodes is selected as 7.

## 3. Results and Discussion

### 3.1. Establishment and Prediction of the Logistic Model of Financial Indicators

#### 3.1.1. Establishing a Logistic Model of Financial Indicators

We add nonfinancial indicator variables and four common factors for the likelihood ratio test, and the specific values are shown in Table 3.

The comprehensive indicator early warning model refers to adding the nonfinancial indicator variable 12 to the pure financial indicators. It is further concluded that the Sig. values are less than 0.05 and pass the significance test. The fitting effect of this model is good.

#### 3.1.2. Comprehensive Index Logistic Model Fitting Test

We use the corporate financial data as test data to test the comprehensive index Logistic model. The results are shown in Table 4. After adding nonfinancial indicators, the obtained comprehensive Logistic model is fitted and tested, and the test results are safe, light, and severe. The prediction accuracy is 90.00%, 80.00%, and 90.00%, respectively, and the overall fitting test result was 87.00%.

Using financial data as forecast data to test the comprehensive index Logistic model, the results are shown in Table 5. The prediction accuracy of the Logistic financial early warning model after adding nonfinancial indicators for safety, light, and severe is 95%, 60.0%, and 80.0%, respectively, and the overall prediction test result is 78.0%.

### 3.2. Model Training and Prediction

After the design and adjustment of the BP neural network model, the training of the sample data is started, so that the network can distinguish the output vector of the financial warning area of the enterprise. In this paper, combined with the number of nodes in the hidden layer above, according to the formula, multiple solutions are performed to obtain multiple values, and the bring-in test is carried out in turn. According to the size of the error, when the hidden layer is 7, the MSE minimum fitting effect is the best. When the number of nodes with layers is set to 7, the sample training error curve is shown in Figure 2.

The training is carried out according to the results of the early warning area of the training sample. According to the comparison between the training value and the actual value in Figure 3, the error between the fitting value and the actual value is not large, and the fitting degree is good. The prediction accuracy of the training value is shown in Table 6.

The predicted test results obtained from the predicted samples are shown in Figure 4.

According to the results of training and equations, it can be judged that when the hidden layer is 7, the fitting effect and prediction effect of the model established in this paper are the best, and the overall test results are 100% and 93%, respectively. The fitting result of the BP neural network can be calculated to be optimal, and the fitting result for the three-year financial warning result of the enterprise reaches 100%. It can be said that when the hidden layer node is set to Table 7, the effect of the model is optimal. The prediction test is then carried out on the financial data of the prediction sample. According to Table 7, it can be seen that the prediction effect is slightly worse than the fitting result. For the mild early warning interval, the overall prediction test result is 93%.

When the number of hidden layer nodes is small, the acquisition ability is poor, the learning speed is slow, and the accuracy rate is relatively low. When the number of nodes increases, the accuracy rate is improved. Therefore, the parameters of the model selected in this paper are detailed in Table 8.

### 3.3. Comparative Analysis of Financial Early Warning Models

Financial early warning research is mainly divided into qualitative and quantitative research. Qualitative research often uses financial professionals to make subjective judgments, but the results are subjective and lack objectivity and fairness. Quantitative research mainly analyzes financial data, reduces the subjectivity of human judgment, and improves the accuracy of prediction through mathematical models.

In practice, financial early warning usually adopts a combination of qualitative and quantitative research methods. Through the methods established by various models, the early warning results are closer to reality and more accurate. Traditional mathematical statistics need to set assumptions and constraints, which cannot fit the reality well, and artificial neural network can better make up for this problem. The comprehensive logistic model with qualitative indicators is not as accurate as the BP neural network. Simple mathematical statistical models have higher requirements on data and more restrictions on the use of models. The correlation between indicators needs to be considered when building models. BP neural network has no constraints on data indicators and has self-learning and feedback capabilities. These advantages have greatly improved the accuracy of financial early warning models.

### 3.4. Establishing a Financial Early Warning System

In recent years, with the continuous changes in the industry, many investors have entered the Chinese market, and the formation of a diversified pattern has also brought huge challenges to Chinese enterprises. The enterprise system is huge and the organizational structure is complex. It is difficult to avoid risks only by relying on the financial early warning model. It is imperative to establish a corresponding early warning system. Chinese enterprises pay more and more attention to the use of scientific methods for management, and managers need to grasp the operating conditions and financial conditions. At this time, the financial early warning has become one of the important management methods to monitor enterprise risks. The financial early warning system can be applied to the business activities of various capital transactions of the enterprise. It is a kind of research based on various financial-related data of the enterprise over the years or peers and makes full use of the theoretical foundations of finance, management, etc. When the enterprise falls into a financial crisis, an early warning signal is issued in time to notify managers to be more vigilant. An excellent financial early warning system suitable for enterprises should include the collection and processing of financial information, supervision, and prevention analysis of financial risks. The collection and processing of data and information is a prerequisite for establishing an early warning system, supervision is the core part, and analysis and response are the keys to risk early warning.

## 4. Conclusion

1. This paper collects the financial indicators of enterprises from 2017 to 2019, and the data mainly come from the stock exchanges and the CCER database. Three criteria are selected as the basis for dividing the early warning degree of energy companies, and the financial data of 40 companies in the same accounting period of 2 years are selected for research, and then the data of 20 companies are selected as prediction test samples for testing.
2. Comparing the Logistic model with the BP neural network, the BP neural network does not have strict requirements on financial indicators in terms of constraints. According to the training results and prediction results, the BP neural network is better than the Logistic model. The calculation of the Logistic model is relatively complex, but it can be expressed in mathematical expressions. BP neural network has strong self-learning ability and computing ability, but it cannot write specific equations. According to the conclusion of the municipal research carried out in this paper, BP neural networks are more suitable for financial early warning of Chinese enterprises.

## Figures and Tables

**Figure 1:** Design steps of financial early warning model.

**Figure 2:** Sample training error curve.

**Figure 3:** Comparison between training and actual data.

**Figure 4:** Comparison between training and actual data.

**Table 1:** Sample data grouping.

Warning interval	Training data	Prediction data	Total
Safety warning zone	40	20	60
Light warning range	20	10	30
Severe warning range	10	5	15
Total	70	35	105

**Table 2:** Financial indicator variables that passed the test.

Number of variables	Indicator name
1	Total operating cost ratio
2	ROA
3	Assets and liabilities
4	Capital adequacy ratio
5	Current ratio
6	Quick ratio
7	Current asset turnover
8	Accounts Receivable Turnover
9	Asset cash ratio
10	Net asset growth rate
11	Financial leverage
12	Audit report

*Note.* Variable 12 is a nonfinancial indicator, the rest are financial indicators.

**Table 3:** Likelihood ratio test table.

Effect	Standard			Likelihood ratio test		
	Simplified model	Simplified model	−2*x* log-likelihood of the reduced model	*K* ^2^	df	Significant level
	A1C	BIC				
Intercept	100.34	129.41	74.32	0	2	0
FAC1_1	129.84	155.67	102.41	24.32	2	0
FAC2_1	174.69	200.31	161.53	74.37	2	0
FAC3_1	70.13	97.95	54.31		2	0
FAC4_1	78.85	100.24	58.51		2	0
12	75.35	97.65	52.46		2	0

**Table 4:** Comprehensive index Logistic model fitting test results.

Observed value	Predicted value			Percent correction (%)
	Safe	Light	Severe	
Safety warning zone	36	4	0	90.00
Light warning range	*3*	16	1	80.00
Severe warning range	0	1	9	90.00
Total percentage	56%	30%	14%	87.00

**Table 5:** Prediction test results of the Logistic model for comprehensive indicators.

Observed value	Predicted value			Percent correction (%)
	Safe	Light	Severe	
Safety warning zone	19	1	0	95.00
Light warning range	*2*	6	2	60.00
Severe warning range	0	1	4	80.00
Total percentage	60%	23%	17%	78.00

**Table 6:** Classification diagram of fitting results.

Observed value	Predicted value			Percent correction (%)
	Safe	Light	Severe	
Safety warning zone	40	0	0	100.0
Light warning range	0	20	0	100.0
Severe warning range	0	0	10	100.0
Total percentage	57.1%	28.6%	14.3%	100.0

**Table 7:** Classification of prediction test results.

Observed value	Predicted value			Percent correction (%)
	Safe	Light	Severe	
Safety warning zone	20	0	0	100.00
Light warning range	*2*	8	0	80.00
Severe warning range	0	0	5	100.00
Total percentage	63%	23%	14%	93

**Table 8:** Parameters of the BP neural network financial early warning model.

Model design	Parameter
Network level	Number of nodes
Input layer	12
Hidden layer	7
Input layer	1
Transfer function	Sigmoid
Training function	Trainlm
Learning rate	0.01
System error	0.001
Number of iterations	100,000

## Data Availability

The data used to support the findings of this study are included in the article.
